# Informative SNP Selection Based on a Fuzzy Clustering and Improved Binary Particle Swarm Optimization Algorithm

**DOI:** 10.1155/2022/3837579

**Published:** 2022-06-16

**Authors:** Zejun Li, Li Ang, Wei Shi, Ning Xin, Min Chen, Hua Tang

**Affiliations:** ^1^School of Computer and Information Science, Hunan Institute of Technology, Hengyang 412002, China; ^2^College of Information Science and Engineering, Hunan University, Changsha, Hunan 410082, China; ^3^Minimally Invasive Thoracic Surgical Center, Shanghai Changzheng Hospital, Navy Military Medical University, Shanghai, China

## Abstract

Single-nucleotide polymorphism (SNP) involves the replacement of a single nucleotide in a deoxyribonucleic acid (DNA) sequence and is often linked to the development of specific diseases. Although current genotyping methods can tag SNP loci within biological samples to provide accurate genetic information for a disease associated, they have limited prediction accuracy. Furthermore, they are complex to perform and may result in the prediction of an excessive number of tag SNP loci, which may not always be associated with the disease. Therefore in this manuscript, we aimed to evaluate the impact of a newly optimized fuzzy clustering and binary particle swarm optimization algorithm (FCBPSO) on the accuracy and running time of informative SNP selection. Fuzzy clustering and FCBPSO were first applied to identify the equivalence relation and the candidate tag SNP set to reduce the redundancy between loci. The FCBPSO algorithm was then optimized and used to obtain the final tag SNP set. The prediction performance and running time of the newly developed model were compared with other traditional methods, including NMC, SPSO, and MCMR. The prediction accuracy of the FCBPSO algorithm was always higher than that of the other algorithms especially as the number of tag SNPs increased. However, when the number of tag SNPs was low, the prediction accuracy of FCBPSO was slightly lower than that of MCMR (add prediction accuracy values for each algorithm). However, the running time of the FCBPSO algorithm was always lower than that of MCMR. FCBPSO not only reduced the size and dimension of the optimization problem but also simplified the training of the prediction model. This improved the prediction accuracy of the model and reduced the running time when compared with other traditional methods.

## 1. Introduction

SNPs describe the genetic diversity caused by the replacement of a single nucleotide in a DNA sequence in 1% or more of a population [1–3]. Although the genotype of all SNP loci could be identified through whole-genome sequencing (WGS), it is costly and sometimes time-consuming to perform [4, 5]. Therefore, there is a need to identify tag SNPs. A tag SNP is a representative SNP in a highly correlated haplotype region. Computational methods can then be used to study complex genetic diseases [6–13], drug targets [14–16], and viral evolution [17–19]. Therefore, the selection of the tag SNPs is becoming increasingly important in current genomic research, and many methods for tag SNP selection have been proposed. These can be divided into three categories: (1) linkage disequilibrium- (LD-) based methods, (2) haplotype block-based methods, and (3) prediction accuracy-based methods.

Linkage disequilibrium describes the occurrence of alleles belonging to two or more gene locations on a chromosome simultaneously, which is higher than the random occurring frequency. The LD-based tag SNP selection method selects a set of tag SNP loci with a high LD among the loci so that the remaining number of untagged SNP loci is still relatively high. This kind of method is often used to classify SNPs of a given region into multiple LD clusters so that the SNPs within the LD cluster end up having a strong correlation (*r*^2^) of 0.8 or higher and hence carrying similar variant information. The algorithm then selects a few representative SNPs among these clusters, which form a tag SNP set [20–23]. The LD-based algorithms are usually fast and are not necessarily limited to haplotype blocks. However, the resulting tag SNP set is not always optimal, and it cannot distinguish all haplotypes within the LD region [24]. In addition, the LD-based method only considers the information associated between the SNP pairs and ignores the association among multiple SNPs and the information from a single SNP locus.

In the haplotype block-based method, genomic sequencing data are divided into several discrete haplotype blocks according to the theory that the number of human haplotypes is far less than the theoretical number [25]. A minimum number of SNP sets within each block need to be identified to enable the SNPs to distinguish every single haplotype in the corresponding block [26, 27]. The haplotype block-based method can resolve some of the LD-based method limitations. For example, the selected tag SNP set can identify most haplotype patterns, with only a small amount of variation information missing. In addition, it reduces the computational complexity on a large scale, facilitating the prediction of large datasets. However, haplotype blocks are challenging to identify as they cannot be defined using a single criterion. The incorrect identification of the haplotype block will result in the identification of false-positive tag SNPs. In addition, haplotype block-based methods for tag SNP selection usually only make use of the relationship between SNP loci within a block while ignoring the relationship between SNP loci outside the block. When there are many independent SNPs in the dataset, the prediction results obtained by this model are usually of poor quality.

In order to overcome the low accuracy of the LD method and the uncertainty of the haplotype block method, Halldorsson et al. proposed an informative SNP locus selection method based on prediction accuracy [28]. This method uses a set of SNP loci known as informative SNPs to reconstruct the remaining nontag SNP loci with high accuracy. The ability of the tag SNPs to represent all other SNPs is generally assessed via the prediction accuracy evaluation index. A higher prediction accuracy indicates an improved ability for the tag SNPs to restore the genotypes of other unlabeled SNPs, eventually improving the efficiency of the research process. Furthermore, to minimize the risk of overfitting the model, the leave-one-cross-validation (LOOCV) method is often used. This method utilizes a *k*-fold cross-validation method whereby *k* is assumed to be equal to the number of samples (*N*). The algorithm then takes one sample as the test set and the other *N*‐1 samples as the training sets. The procedure is repeated *N* times, and the average accuracy (ACC) is used to estimate the population-wise accuracy according to the following formula:

(1) $$\begin{array}{c} \text{Acc}=1-\frac{\sum_{i}^{N}\sum_{j}^{\left|O\right|}\left|s_{j}-s_{j}^{\prime }\right|}{\left|O\right|\times N}, \end{array}$$

In this formula, *O* represents the set of nonlabel SNPs, |*O*| represents the number of nonlabel SNPs, *N* represents the sample size, *s*_*i*_ represents the observed SNP locus genotype in the sample, *s*_*i*_′ represents the locus genotype output by the prediction model, and the absolute value of the difference between the two represents the prediction error. Note that this formula applies only to the genotype from a haploid species (haplotype) since the nonlabeled SNP prediction problem can only be expressed using a classification of 0 and 1. However, the genotype in other species is usually encoded as 0, 1, and 2. This may result in an accuracy greater than one making the result meaningless.

An alternative approach is to identify a set of informative SNP loci that can accurately predict the residual noninformation SNP loci (nontag SNPs) and reconstruct the corresponding haplotype sequence. Therefore, Halperin et al. proposed the tag SNP method to maximize prediction accuracy (STAMTA) for genotyping samples from a group of unrelated individuals [29]. Although the existing tag SNP selection methods improve the prediction accuracy of SNP sites under certain conditions, they are far from enough for practical applications. These methods still have some limitations, including long calculation time, high complexity, low precision, and unclear biological significance. Due to the existence of these problems, the information-rich SNP site selection and its accuracy prediction are still challenging in genome research. In order to overcome this problem, the particle swarm optimization algorithm (PSO) can be used to optimize the characterization of SNP data by improving the prediction accuracy without increasing the calculation time. Because PSO has better optimization performance for complex optimization problems. This method involves using the linkage disequilibrium between SNPs to cluster all SNPs and construct sets of candidate tag SNPs. Then, a candidate set of tag SNPs is optimized and selected based on an improved particle swarm algorithm of the bionic algorithm, thus selecting the informative SNPs. Finally, the support vector machine (SVM) model is used to predict the nontag SNPs and reconstruct the haplotype. Specialized software and the radial basis function (RBF) kernel are then used to identify the C-SVC model in SVM. The gamma and loss parameters of the kernel function are obtained using a grid search of 0.07 and a cross-validation accuracy of 7. This method does not rely on the partitioning of haplotype blocks and makes full use of the characteristics of the tag SNP selection to design an appropriate fitness function. The resulting model is therefore a less complex and more accurate algorithm with a shorter computation time.

In order to overcome the above-mentioned shortcomings and deficiencies of the existing work, we aimed to evaluate the impact of using a newly developed optimized fuzzy clustering binary particle swarm optimization algorithm (FCBPSO) on the SNP selection accuracy and algorithm running time in comparison with traditional SNP selection algorithms.

## 2. Materials and Methods

### 2.1. Description of the Tag SNP Selection Problem

The tag SNP selection problem was defined in a sample set of *n* chromosomes, whereby each chromosome contains *m* SNP loci expressed as

(2) $$\begin{array}{c} H=\left\{h_{1},h_{2},\cdots ,h_{n}\right\},\\ h_{i}=\left\{{\text{SNP}}_{1},{\text{SNP}}_{2},\cdots ,{\text{SNP}}_{m}\right\}. \end{array}$$

For convenience, we only considered haploid organisms so that each chromosome can be expressed as a binary string of 0 and 1, and all DNA samples were expressed as a matrix (*M*) of size *n* × *m*. The SNP at the *j*^th^ locus in chromosome *i* is represented using the formula

(3) $$\begin{array}{c} M\left[i,j\right]\in \left[0,1,-\right], \end{array}$$

where 1 represents major alleles, 0 represents minor alleles, and “−” represents the missing locus.

Our goal was to find a tag SNP locus set *R* from the given sample set *H* so that the number of elements in *R* is as small as possible and the prediction accuracy of the nontag SNPs is as high as possible. Informative SNP selection has been proven to be an NP-hard problem. Therefore to find an optimal solution, our method mainly consisted of two parts. The first part involved the use of fuzzy clustering (FC) to obtain the candidate informative SNP set. In the second part, the particle swarm optimization (PSO) algorithm was used to identify the informative SNP set. These two methods are described in detail below.

### 2.2. Application of the FC Algorithm to Identify the Candidate Informative SNP Set

The FC theory was first proposed in 1965 by Zadeh and is now widely used in various fields [30, 31]. The 2 main advantages of FC are the flexible use of distance and the ability to incorporate some known membership values into the numerical optimization. This method could be applied in our study to identify the candidate tag SNP sets as the LD relation among SNPs satisfied the symmetry and reflexivity criteria. This clustering method is efficient and convenient since there is no need to set the clustering number in advance. The following formula was therefore used to identify the LD relationship. Assuming that A(a) and B(b) are the major (minor) alleles at two SNP loci, then the LD between the two loci can be calculated as

(4) $$\begin{array}{c} \;D=f_{AB}-f_{A}\times f_{B}. \end{array}$$

If *D* > 0,

(5) $$\begin{array}{c} \text{LD}=\frac{D}{\min\left(f_{A}\cdot f_{b},f_{a}\cdot f_{B}\right)}. \end{array}$$

If *D* < 0,

(6) $$\begin{array}{c} \text{LD}=\frac{D}{\min\left(f_{A}\cdot f_{B},f_{a}\cdot f_{b}\right)}, \end{array}$$

where *f*_*X*_ signifies the probability of *X* appearing in the group.

For convenience, we assumed that *r*_*ij*_ represents the LD value between the *i*^th^ SNP and the *j*^th^ SNP. Therefore the relationship matrix of the *m* tag SNPs could be defined as *R* = (*r*_*ij*_)_*m*×*m*_ whereby the domain *U* represents the SNP locus. *R* was converted into a fuzzy equivalence relation matrix and clustered using FC since it satisfied the reflexivity and symmetry criteria and had a fuzzy binary relationship with the *U* domain. Therefore, contrary to the traditional flat method, the Warshall algorithm was applied to find the transitive closure of the fuzzy similarity matrix and obtain the fuzzy equivalence relation matrix *t*(*R*) to reduce the computational complexity and time [32]. After obtaining *t*(*R*), the Boolean matrix *t*(*R*)_*λ*_ of the fuzzy equivalence relation was obtained according to the preset *λ* parameters, by which the equivalence class [*I*]_*R*_ was calculated. The calculation was performed according to Formula (7). Finally, the candidate tag SNP *SR* set was obtained by calculating the center of each equivalence relation class.

The process used to obtain the candidate tag SNP set was calculated in five steps according to the equivalence relation described below.

**Algorithm 1 .**

Input: an *n*∗*m* chromosome sample matrix *M*, parameters *λ* ∈ [0, 1.]
Output: a candidate tag SNPs set SI
Step 1: the fuzzy similarity matrix of the matrix *M* was calculated using Formulas (4)–(6)
Step 2: the transitive closure of the similarity matrix *R* was calculated using the Warshall algorithm, and the fuzzy similarity relation matrix was transformed into the fuzzy equivalence relation matrix
Step 3: the fuzzy equivalence relation matrix *t*(*R*) was transformed into a fuzzy equivalence Boolean matrix *t*(*R*)_*λ*_ according to the preset parameters *λ*, and then, the equivalence relation class [*I*]_*R*_ was calculated. The division method of the equivalence relation class is as shown in Formula (7):
  (7) $$\begin{array}{c} t\left(R\right)=\overset{¯}{{\left(r_{ij}\right)}_{m\times m}},\\ t{\left(R\right)}_{\lambda }=\left(\overset{¯}{r_{ij}{\left(\lambda \right)}_{m\times m}}\right)=\left\{\begin{array}{c} 0,r_{ij}<\lambda ,\\ 1,r_{ij}\geq \lambda , \end{array}\right. \end{array}$$
  where ∀*SNP*_*i*_, *SNP*_*j*_ ∈ *S*, if (*r*_*ij*_(*λ*)) = 1, *SNP*_*i*_, and *SNP*_*j*_ belong to the same equivalence relation class
Step 4: the center of each equivalence relation class was calculated, and each class center was combined into the candidate tag SNP set SI. The center of each class was obtained by calculating the sum of the LD value of each locus and other members in the class. The largest locus was regarded as the class center.

### 2.3. Development of the PSO Algorithm

#### 2.3.1. The Theoretical Principle behind the Improved PSO Algorithm

PSO was derived from the predation behavior of flocks and was first proposed by Dr. Eberhart and Dr. Kennedy in 1995 [33]. The original PSO algorithm concept provided a simple solution to each optimization problem by regarding it as a bird searching space, called “particle,” whereby each particle flies at a certain speed. When each particle moves in the search space, it needs to consider its current optimal historical position (pbest) and the current searched optimal historic population position (gbest). The optimal position of the particles is evaluated for fitness, using the objective function. Optimality means the highest fitness, and in the PSO algorithm, it means that the birds in the flock find the most food at a particular location. After an iterative cycle, the particles of the whole group move towards the optimal solution, like birds foraging for food. Due to the simplicity of the PSO algorithm and its good optimization ability, it is improved and used for optimization.

#### 2.3.2. Application of the Improved PSO Algorithm

In this study, we assumed that for a population size of *m* particles, each particle has *n* dimension space target search. This was defined with the equations *V*_*i*_ = (*v*_*i*1_, *v*_*i*2_, ⋯, *v*_in_) whereby *i*^th^ is the particle speed and *X*_*i*_ = (*x*_*i*1_, *x*_*i*2_, ⋯, *x*_in_) is the current location of the *i*^th^ particle. The location of the optimal solution currently found by particle *i* is *P*_*i*_ = pbest_*i*_ = (*p*_*i*1_, *p*_*i*2_, ⋯⋯⋯*p*_in_), and therefore, in the (*t* + 1)^th^ generation, the speed update formula of the *i*^th^ particle in the *d*(1 ≤ *d* ≤ n) dimension is as shown in Equation (8), and the displacement update formula is as shown in Equation (9):

(8) $$\begin{array}{c} v_{id}\left(t+1\right)=wv_{id}\left(t\right)+c_{1}\mathrm{rand}\left(\right)\left[p_{id}\left(t\right)-x_{id}\left(t\right)\right]+c_{2}\text{Rand}\left(\right)\left[g_{id}\left(t\right)-x_{id}\left(t\right)\right], \end{array}$$

(9) $$\begin{array}{c} x_{id}\left(t+1\right)=x_{id}\left(t\right)+v_{id}\left(t+1\right). \end{array}$$

In these equations, *w* is the inertia factor, representing the inheritance of the velocity of the original particle and reflecting the motion inertia of particles. *c*_1_ and *c*_2_ are the two acceleration constant factors, representing the tendency of particles moving towards their historical best position and the optimal position of the group, which belongs to the cognition of themselves and the society. rand() and Rand() are two random functions between the values of [0, 1]. To avoid particles that are beyond the boundary of the search space, *v*_*id*_ was limited to a certain range, that is, *v*_*id*_ ∈ [−*v*_*id* max_, *v*_*id* max_].

The general steps followed in the development of the PSO algorithm were as follows.

#### 2.3.3. Development of the Binary Particle Swarm Optimization (BPSO)

The general PSO algorithm is often applied to the postgroup domain optimization problem due to its simplicity and fast convergence speed. However, its further development is limited because it only applies to the functional domain of continuous space. To solve this problem, Kennedy and Eberhart improved it in 1997 and proposed the binary particle swarm optimization (BPSO) algorithm for discrete space [34]. Note that lots of improved version of PSO have been proposed for various applications [35–37].

In the new BPSO algorithm, the coding mode terms were modified so that the velocity no longer represents the rate of positional change but instead represents the quantity probability reference of the particle positional change, which allows the position to be expressed as a discrete type. After the velocity particle updates according to Formula (8), the sigmoid function was used as shown in Formula (10) to map its velocity value to the interval of [0,1]. The particle position was then updated according to Formula (11) to discretize its position, thus applying the BPSO algorithm successfully to the discrete space field.

(10) $$\begin{array}{c} Sig\left(v_{id}\right)=\frac{1}{1+\exp\left(-v_{id}\right)}, \end{array}$$

(11) $$\begin{array}{c} x_{id}=\left\{\begin{array}{cc} 1, & \text{sig}\left(v_{id}\right)\geq \mathrm{rand}\left(\right),\\ 0, & \text{else}. \end{array}\right. \end{array}$$

Formula (11) was then used to transform the sigmoid function to calculate the probability that the particle takes the value of 1 at the position.

There are some issues in applying the traditional BPSO algorithm directly to the selection of informative SNPs. For example, if the new particle swarm produces more particles than the initial number of tag SNPs given in advance, the unqualified solution problem occurs. In addition, when the BPSO algorithm searches for the optimal solution, the particle should be closer to the current to find the optimal particle in the later stage of its iteration. Therefore, the speed of the forward-moving particles during this time is gradually slowed to almost zero. In other words, the factors that affect the particle speed should be just “self-cognition” *c*_1_∙rand()∙(pbest_*id*_ − *x*_*id*_) and “social cognition” *c*_2_∙rand()∙(gbest_*id*_ − *x*_*id*_).

In order to overcome this problem, a revision strategy was applied to the solution. When the number of tag SNPs was larger than the number of given tag SNPs, the reduction correction strategy was adopted. Conversely, when the number of tag SNPs was less than the preset number, the increase correction strategy was adopted. For example, if the number of SNPs of a given tag was six and a newly generated particle had a code of “010100110010111,” the particle would therefore select the second, fourth, seventh, eighth, eleventh, thirteenth, fourteenth, and fifteenth SNP loci, and a total of eight SNPs would be used as tag SNPs. Therefore, a reduction correction strategy was adopted for such cases. The applied corrective measures were defined as follows.

If the number of pregiven tag SNPs is *S*, for the *i*^th^ particle, |*Xi*| = (*x*_*i*1_, *x*_*i*2_, ⋯, *x*_|*SI*|_). The optimization process is still based on the SI candidate set of the tag SNPs so that the dimension of the *i*^th^ particle is equal to the number of candidate tag SNPs, assuming |*X*_*i*_| represents the number of tag SNPs selected across the *i*^th^ label particle, of which the value is equal to the number of codes whose value is 1. *clu*_*kj*_ indicates the class *k* to which the first candidate SNP locus belongs, |*clu*_*kj*_| indicates the size of the *k*^th^ cluster, and the size of |*clu*_*kj*_| reflects the ability of the *j*^th^ candidate SNP to represent other loci. The larger the |*clu*_*kj*_|, the higher the probability that the other loci information is contained in the candidate tag SNPs, and therefore more likely, the candidate tag SNPs can represent other SNP loci.

If *S* < |*X*_*i*_|, a corrective reduction strategy was adopted to sort the SNP locus, whereby *X*_*ij*_ = 1, according to the size of |*clu*_*kj*_|, keeping the first *S* tag SNP, and encoding the following (|*X*_*i*_| − *S*) loci from 1 to 0.

If (|*X*_*i*_| − *S*), a corrective reduction strategy was adopted to sort the SNP locus, whereby *X*_*ij*_ = 0, according to the size of |*clu*_*kj*_| and encoding the previous (*S* − |*X*_*i*_|) candidate tag SNPs from 1 to 0.

For the second problem mentioned above, the updated formula of the traditional BPSO algorithm was improved as shown in

(12) $$\begin{array}{c} v_{id}\left(t+1\right)=c_{1}\mathrm{rand}\left(\right)\left[p_{id}\left(t\right)-x_{id}\left(t\right)\right]+c_{2}\text{Rand}\left(\right)\left[g_{id}\left(t\right)-x_{id}\left(t\right)\right]. \end{array}$$

The advantage of Formula (12), when compared with Formula (8), is that it removes the inheritance of the previous particle-generated velocity by only updating the velocity determined by “self-cognition” and “social cognition.” This slows down the forward-moving velocity of the particle and makes it easier for the particle to approach the current optimal solution being searched, avoiding the phenomenon of skipping over the optimal solution. Further analysis of the situation is described below.

The values of (pbest_*id*_ − *x*_*id*_) and (gbest_*id*_ − *x*_*id*_) can only be 1, 0, and -1.

If the value is 0, then it is likely to be pbest_*id*_ = *x*_*id*_ or gbest_*id*_ = *x*_*id*_.

If the value is 1, then it is likely to be pbest_*id*_ = 1 or gbest_*id*_ = 1 and *x*_*id*_ = 0.

If the value is -1, then it is likely to be pbest_*id*_ = 0 or gbest_*id*_ = 0 and *x*_*id*_ = 1.

Given the above, the velocity *v*_*id*_ can be greater than, less than, or equal to zero.

If the velocity *v*_*id*_ = 0, that is, pbest_*id*_ = *x*_*id*_ or gbest_*id*_ = *x*_*id*_, then the value of the particle at the d dimension is the same as the optimal position of the current particle or the optimal historical position of the particle, and the locus should not change.

If the velocity *v*_*id*_ < 0, that is, pbest_*id*_ = 0 or gbest_*id*_ = 0 and *x*_*id*_ = 1, then the value of the particle at the *d* dimension is unequal to the optimal position of the current particle or the optimal historical position of the particle, and the locus is more likely to change from 1 to 0.

If the velocity *v*_*id*_ > 0, that is, pbest_*id*_ = 1 or gbest_*id*_ = 1 and *x*_*id*_ = 0, then the value of the particle at the *d* dimension is unequal to the optimal position of the current particle or the optimal historical position of the particle, and the locus is more likely to change from 0 to 1.

Based on the above analysis, the change of particle position evaluation and the change of the velocity consistent, in Formula (10), were further improved as shown in

(13) $$\begin{array}{c} \text{Sig}\left(v_{id}\right)=\left\{\begin{array}{c} 1-\frac{2}{1+\exp\left(-v_{id}\right)},\text{if }v_{id}<0,\\ \frac{2}{1+\exp\left(-v_{id}\right)}-1,\text{if }v_{id}>0. \end{array}\right. \end{array}$$

Formula (13) coincided with the above speed analysis and position update changes. When speed *v*_*id*_ = 0, the improved probability mapping function takes a value of 0, and when *v*_*id*_ < 0, or *v*_*id*_ > 0, its mapped value tends to be 1.

According to the analysis above, when the iteration reaches a later stage, the displacement formula also changes, and the particle position formula was therefore updated as shown in

(14) $$\begin{array}{c} x_{id}\left(t+1\right)=\left\{\begin{array}{c} 0,\\ 1, \end{array}\begin{array}{c} \text{ Sig}\left(v_{id}\left(t+1\right)\right)\geq \mathrm{rand}\left(\right),\\ \begin{array}{cc} \; & \text{else} \end{array}, \end{array}\right.\text{ if }v_{id}\left(t+1\right)<0, \end{array}$$

(15) $$\begin{array}{c} x_{id}\left(t+1\right)=\left\{\begin{array}{c} 1,\\ x_{id}\left(t\right), \end{array}\begin{array}{c} \begin{array}{cc} \; & \text{Sig}\left(v_{id}\left(t+1\right)\right)\geq \mathrm{rand}\left(\right), \end{array}\\ \begin{array}{cc} \; & \text{else} \end{array}, \end{array}\;\right.\text{if }v_{id}\left(t+1\right)>0. \end{array}$$

Formula (14) shows that in the case of a velocity *v*_*id*_(*t* + 1) < 0, the smaller *v*_*id*_(*t* + 1) is larger, and the current position of the particle is more likely to be converted to 0; otherwise, it does not need to be changed. In the case that *v*_*id*_(*t* + 1) > 0, the larger *v*_*id*_(*t* + 1) is larger than sig(*v*_*id*_(*t* + 1)), and the current particle position is more likely to be converted to 1; otherwise, it means that the *x*_*id*_(*t* + 1) is equal to 0, and the locus at that position does not need to be updated. Therefore, through these improvements, the particle can more easily approach the optimal global particle. When the velocity is 0, the probability of the particle locus equaling 0 increases.

#### 2.3.4. Optimization Based on the Improved BPSO

The BPSO algorithm was optimized as follows.

*(1) Population Initialization*. Similar to other bionic optimization algorithms, the start of the BPSO optimization process is initialization. The initialization of the BPSO always requires the initialization and assignment of velocity values to each particle except for the initial particle swarm generation. Suppose the candidate set generated by fuzzy clustering is SI. In that case, the initialization requires a binary coding of the SI set whereby 1 means a locus label, 0 means a nontag locus, and the initial particle swarm is randomly generated. The initial velocity of each particle is randomly initialized according to Formula (16):

(16) $$\begin{array}{c} v_{id}\left(0\right)=v_{\min}+\mathrm{rand}\left(\right)\left(v_{\max}-v_{\min}\right), \end{array}$$

where *v*_min_ and *v*_max_ represent the minimum and maximum values of the particle speed, respectively. The algorithm is then updated according to Formula (8) in the early stage of the iteration based on the initial particle velocity. While in the late iteration stage, the algorithm is updated according to Formula (12) to let the particle get closer to the current optimum.

*(2) Designing the Fitness Function*. The particle that has the memory function was initialized by the pbest and gbest particles in the search process so that the particles can reach the approximate optimal solution more quickly. pbest and gbest were selected according to the particle fitness. Since the number of tag SNPs contained within the particles was consistent, the design of the fitness function does not need to consider the number of tag SNPs, and therefore, it is possible to calculate the fitness of particle *X* according to

(17) $$\begin{array}{c} f\left(X\right)=\frac{1}{m}\overset{\left|X\right|}{\underset{j=0}{\sum }}\left|clu_{kj}\right|,j\in \left[1,m\right]. \end{array}$$

From Formula (17), the fitness of a particle can be determined by the number of other loci represented by the selected tag SNPs in its particles. The ability of each tag SNP to contain information of other loci is determined by the size of the class to which it belongs. The pbest particle search provides the best solution among the solutions in the current search, that is, the one with the highest fitness. Conversely, the gbest search provides the optimal current solution for all particles. This means that pbest and gbest need to be updated in each iteration.

The FCBPSO method improves the BPSO tag SNP selection method based on FC. The FC algorithm utilizes the equivalent relation clustering to identify and optimize the set of candidate tag SNPs. Then, the BPSO algorithm is applied to select the tag SNPs. Finally, the nontag SNPs are estimated by using the tag SNPs with the SVM classification algorithm. The method flow chart is shown in Figure 1, and the basic process is shown below:

The flow chart of its algorithm steps is shown in Figure 1.

### 2.4. Evaluation of the New FCBPSO

To validate the effectiveness of our method, we compared FCBPSO for tag SNP selection in the bionic algorithm [38], SPSO [39], and MCMR methods [40]. Liao et al. proposed an NMC tag SNP selection method based on the ant colony algorithms in 2012. The method utilized a mean clustering algorithm in the sample reconstruction stage, with the accuracy of the sample reconstruction as the optimization target, and then solved by the ant colony algorithm. In the SPSO selection method, all SNP loci are encoded by using the discrete BPSO. The design of the fitness function mainly considers the number of tag SNPs and their prediction accuracy according to the *k*-nearest neighbor method. In the MCMR method, the principle of maximum association and minimum redundancy between SNPs is used to select tag SNPs. The MCMR method can be applied to different platforms and large datasets, but it is complex and time-consuming to perform.

Experimental data were obtained from the actual datasets ENm013, ENr112, and ENr113 published by HapMap. These datasets were sampled from 30 CEPH families, which belong to regions containing SNP loci on chromosome 7q21.13. The basic information of each dataset is shown in Table 1.

The tag SNP set was selected in FCBPSO, and the SVM model was used to predict the nontag SNPs. Two evaluation indexes, prediction accuracy and computational time, were used in the comparison experiment. The computational tests were carried out on a personal computer with a Pentium IV processor and 4 GB RAM.

## 3. Results

### 3.1. Prediction Accuracy

The prediction accuracy of the newly developed FBBPSO, NMC, SPSO, and MCMR is shown in Figure 2.

As shown in Figure 2, in most cases, the prediction accuracy of the FCBPSO algorithm is higher than that of the other algorithms. In Figures 2(a) and 2(b), when the number of tag SNPs was low, the prediction accuracy of FCBPSO was slightly lower than that of MCMR. However, as the number of tag SNPs increased, FCBPSO had the highest prediction accuracy, followed by MCMR. When the number of tag SNPs reached 10, the prediction accuracy of FCBPSO exceeded 98%, while SPSO had a lower prediction accuracy. For the ENr113 dataset, FCBPSO also showed similar superior performance. It is interesting to note that the NMC algorithm could not directly operate on the ENr113 dataset due to the long running time and therefore could not provide any result. As can be seen in Figure 2, the selected tag SNP set by FCBPSO was more informative than those selected by the other three methods and could represent all SNP loci to a greater extent, hence improving the efficiency of subsequent association analyses. In addition, as the number of loci in the sample data increased, the prediction accuracy of the four methods was generally reduced. For example, when 10 SNP tags were selected, the prediction accuracy of FCBPSO for the ENm013 dataset reached 98.7%, but for the ENr113 dataset, the prediction accuracy was only 95.2%. As expected, as the number of the sampled loci increased, a larger number of nontag SNPs with the same number of tag SNPs need to be predicted, and therefore, the prediction error rate will also increase.

### 3.2. Running Time

To further prove the superiority of FCBPSO, we also evaluated the algorithm running time. The prediction accuracy of MCMR was similar to that of FCBPSO and superior to that of other methods. Prediction accuracy is the most important factor when evaluating algorithm performance, as an erroneous judgment of an SNP locus genotype may lead to errors in disease correlation and drug analyses. Therefore, only FCBPSO and MCMR were compared in the run time comparison test. The results are shown in Table 1, and the time unit is second.

As illustrated in Table 2, the running time of FCBPSO is much less than that of MCMR. MCMR uses the postdeletion algorithm to remove redundant SNPs during the construction of the tag SNP subset. In the deletion process based on the candidate tag SNPs, an exhaustive method was used to enumerate each possible informative SNP. Only one redundant SNP site was deleted at a time, and during each iteration, the SVM prediction algorithm was used for both training and testing, which is time-consuming. The FCBPSO method increases the construction velocity of the label SNP subset and updates the position of the formula so that the particle swarm can converge to the optimal solution at a faster rate. Furthermore, the gbest particle used in the prediction model only conducts training and prediction for the optimal global individuals, eventually reducing the running time.

## 4. Conclusion

In this study, we proposed an informative SNP selection method to improve the prediction accuracy of SNP detection and reduce the running time. An FC algorithm based on the equivalence relation was first used to identify a set of candidate tag SNPs. Subsequently, an improved BPSO algorithm was used to optimize the selection of the candidate set of tag SNPs. Different speeds and positions during the pre- and postiteration stages were used to update the formulas, improve the algorithm's convergence speed, and reduce the running time. In the selection process, we adopted a series of measures to improve the performance of the algorithm. The Warshall's method was initially adopted to calculate the transitive closure to obtain the equivalent relation matrix, which has a higher performance when compared with traditional flat methods. Then, the candidate SNP set for the particle swarm initialization process was identified to reduce the size and dimension of the optimization problem. Our final prediction model only needed to provide training to the optimal global individuals in the particle swarm and not repeatedly as in other traditional selection methods based on prediction accuracy. This reduced the running time and improved the efficiency of the model when compared with other traditional methods. In the future, we will integrate other feature selection methods like L0 [41], ridge regression [42], and elastic-net [14, 43] and other computational models like random forest[44, 45] and deep learning [46] to further improve the performance of our prediction model. In addition, this article is limited at discussing a single objective. In fact, there are multiobjectives that need to be considered at the same time, so we will further discuss the situation of multioptimization objectives in the future.

## Figures and Tables

**Figure 1:** FCBPSO algorithm flow chart.

**Figure 2:** Comparison of prediction accuracy. (a) The precision accuracy results of the NMC, SPSO, MCMR, and FBPSCO algorithms for the ENm013 dataset. (b) The precision accuracy results of the NMC, SPSO, MCMR, and FBPSCO algorithms for the ENm112 dataset. (c) The precision accuracy results of the SPSO, MCMR, and FBPSCO algorithms for the ENm113 dataset.

**Algorithm 1:** PSO.

**Algorithm 2:** FCBPSO.

**Table 1:** The size of experimental datasets.

Name	Number of SNPs	Number of samples
ENm013	360	120
ENr112	411	120
ENr113	514	120

**Table 2:** Running time comparison of the MCMR and FCBPSO algorithms for the ENm013, Enr112, and ENr113 datasets.

No.	ENm013		ENr112		ENr113	
	MCMR	FCBPSO	MCMR	FCBPSO	MCMR	FCBPSO
2	11100	22.61	3100	20.81	19500	39.59
4	11000	17.51	3000	30.46	18000	53.34
6	10300	16.69	2700	30.75	17000	59.06
7	9600	18.64	1500	34.33	14800	57.22
10	8600	17.56	800	35.97	12000	58.16

## Data Availability

The data are available from the authors on reasonable request.
